The article "Application of Tivantinib for Hepatocellular Carcinoma: A Meta-Analysis Study" was published in 2022. Journal: Evid Based Complement Alternat Med.

# Application of Tivantinib for Hepatocellular Carcinoma: A Meta-Analysis Study

**DOI:** 10.1155/2022/1976788

**Published:** 2022-06-07

**Authors:** Guang-li Luo, Bian-qin Guo, Li-xiang Wu, Yan-xi Shen, Tingting Xie

**Affiliations:** ^1^Key Laboratory for Biorheological Science and Technology of Ministry of Education (Chongqing University), Chongqing University Cancer Hospital, Chongqing 400044, China; ^2^Chongqing Medical University, Chongqing, China

## Abstract

**Objectives:**

The efficacy of tivantinib may have some potential in treating MET-high hepatocellular carcinoma, and we aim to compare tivantinib with placebo for the treatment of MET-high hepatocellular carcinoma.

**Methods:**

Several databases including PubMed, Cochrane Library, Web of Science, EBSCO, and EMbase have been systematically searched through March 2022, and we included studies regarding the treatment of MET-high hepatocellular carcinoma by using tivantinib versus placebo.

**Results:**

We finally include three RCTs. In comparison with placebo for MET-high hepatocellular carcinoma, tivantinib reveals no significant influence on overall survival (*P*=0.21), progression-free survival (*P*=0.13), time to progression (*P*=0.38), or grade ≥3 anemia (*P*=0.50) but increases the incidence of grade ≥3 neutropenia (*P*=0.04).

**Conclusions:**

Tivantinib may provide no additional benefits for MET-high hepatocellular carcinoma.

## 1. Introduction

It is widely accepted that hepatocellular carcinoma results in poor prognosis [1]. Advanced hepatocellular carcinoma leads to poor prognosis [2]. Currently, antiangiogenic drugs and immune checkpoint inhibitor nivolumab have been approved for advanced hepatocellular carcinoma [3]. Although these drugs have some potential in improving median time to progression and overall survival, effective second-line therapies are required for these patients [4].

MET has been found to promote tumour development and metastasis by binding to hepatocyte growth factor (HGF) [5]. One small-molecule MET receptor tyrosine kinase inhibitor, tivantinib has the ability to promote the apoptosis of MET-positive tumour cell lines [6]. MET is thought to be a negative prognostic factor, and tumour tissues after sorafenib therapy have increased overexpression of MET [7, 8]. Tivantinib was reported to inhibit the progression of hepatocellular carcinoma in patients with hepatocellular carcinoma (*P*=0.03) [9].

Several studies have explored the application of tivantinib for MET-high hepatocellular carcinoma, with conflicting results [10]. This meta-analysis is performed to investigate the efficacy of tivantinib for MET-high hepatocellular carcinoma.

## 2. Methods

### 2.1. Study Selection and Data Collection

Several databases including Cochrane Library, PubMed, Web of Science, EBSCO, and EMbase have been systematically searched through March 2022, and we use the search terms “tivantinib” and “hepatocellular carcinoma”. Inclusion criteria are as follows: (1) patients are diagnosed as MET-high hepatocellular carcinoma, (2) treatments are tivantinib versus placebo, (3) outcomes should include overall survival, and (4) only RCT design is involved. We exclude patients with the history of HIV infection or liver transplantation.

### 2.2. Data Extraction and Outcomes

Two investigators extract the same information such as first author, patient number, age, female, Eastern Cooperative Oncology Group (ECOG) performance status, *α*-fetoprotein (AFP) > 200 ng/mL, and detailed methods of two groups.

Overall survival is regarded as the primary outcome. Secondary outcomes are time to progression, progression-free survival, grade ≥3 neutropenia, and anemia. Progression-free survival indicates the time from randomization to the date of first disease progression or death. Time to progression is the time from randomization to the date of the first disease progression [11]. Neutropenia grade is determined using the National Cancer Institute's Common Toxicity Criteria [12]. Anemia grade is classified by National Cancer Institute (NCI) Criteria [13].

### 2.3. Evaluation for Risk of Bias

The risk of bias tool mainly includes performance bias, attrition bias, selection bias, reporting bias, detection bias, and other potential sources of bias [14]. They are used to evaluate paper quality which is ranked as low, unclear, or high [15].

### 2.4. Statistical Analysis

We assess RR or HR with 95% CI for outcomes. Heterogeneity is assessed by I^2^ statistic, and its value more than 50% suggests substantial heterogeneity [16]. The random-effect model is used for all meta-analysis. We also calculate a prediction interval of the overall effect sizes [17]. We conduct sensitivity analysis by omitting one study in turn for the analysis. The difference with *P* < 0.05*P* < 0.05 is statistically significant.

This meta-analysis was based on previously studies, so ethical approval and patient consent were not needed. It was conducted based on Preferred Reporting Items for Systematic Reviews and Meta-Analysis statement and Cochrane Handbook for Systematic Reviews of Interventions [18]. Review Manager version 5.3 is applied for the meta-analysis.

## 3. Results

### 3.1. Search and Characteristics of Studies

Figure 1 showed the detail procedures of study search and selection. We initially found 395 publications and 126 duplicates were removed. Then, 264 papers were excluded after screening titles (*n* = 85) or abstracts (*n* = 179). Two studies were removed because of the same patient samples after reading the full articles and three RCTs were ultimately included [10]. The total sample size of included patients was 572. Among the RCTs included, two studies report tivantinib 120 mg twice daily [19], and the remaining study reports tivantinib 360 mg and then 240 mg twice daily (Table 1) [9]. Three studies report progression-free survival and overall survival [10], two studies report time to progression [20], and two studies report grade ≥3 neutropenia and anemia [19].

### 3.2. Risk of Bias

Figure 2 demonstrates the risk of bias. Among the three included RCTs, one study has unclear risk of randomization [21] and three studies have unclear risk of blinding [10], but all included studies have high quality.

### 3.3. Primary Outcome: Overall Survival

Tivantinib does not substantially affect overall survival (HR = 0.78; 95% CI = 0.52 to 1.15; *P*=0.21) for MET-high hepatocellular carcinoma in comparison with placebo, but significant heterogeneity is seen (I^2^ = 64%, heterogeneity *P*=0.06, Figure 2).

### 3.4. Sensitivity Analysis

Significant heterogeneity is observed. Thus, 95% prediction interval of overall survival is calculated, and it ranges from −1.24 to 2.80, which also shows no statistical difference between two groups. In addition, the study conducted by Santoro et al. may cause the heterogeneity (Figure 2). After excluding this study, tivantinib still did not affect the incidence of overall survival (HR = 0.93; 95% CI = 0.75 to 1.15; *P*=0.51; Figure 3), and no evidence of heterogeneity is observed (I^2^ = 0%).

### 3.5. Secondary Outcomes

Comparised with placebo for MET-high hepatocellular carcinoma, tivantinib does not affect progression-free survival (HR = 0.77; 95% CI = 0.55 to 1.08; *P*=0.13; Figure 4) or time to progression (HR = 0.71; 95% CI = 0.33 to 1.52; *P*=0.38; Figure 5). In the case of adverse events, tivantinib results in the increase in grade ≥3 neutropenia (RR = 11.28; 95% CI = 1.11 to 115.08; *P*=0.04; Figure 6) but has no impact on the incidence of grade ≥3 anemia (RR = 2.83; 95% CI = 0.14 to 56.60; *P*=0.50; Figure 7).

## 4. Discussion

MET-high hepatocellular carcinoma commonly results in poor prognosis, but tivantinib treatment may have the potential in improving its overall survival [11]. This study aims to find the efficacy of tivantinib, and the results reveal no benefits for MET-high hepatocellular carcinoma in terms of progression-free survival, survival, or time to progression after the treatment of tivantinib.

Considering these negative results, several reasons may account for them. Firstly, MET expression may be not associated with the resistance to sorafenib in advanced hepatocellular carcinoma. Secondly, tivantinib may be not the effective MET inhibitor. Thirdly, there is lack of persistent MET activation after sorafenib therapy in advanced hepatocellular carcinoma [11]. In addition to tivantinib, other drugs such as everolimus and ramucirumab also reveal no obvious efficacy for advanced hepatocellular carcinoma [22].

During the sensitivity analysis, we find no heterogeneity after excluding one study [9]. Among the included RCTs, one study involves tivantinib 240 mg twice daily [9], and the other two studies report tivantinib 120 mg twice daily [19]. Tivantinib 240 mg twice daily can provide the additional improvements in progression-free survival and overall survival in MET-high hepatocellular carcinoma, while tivantinib 120 mg twice daily shows no clinical benefits. Thus, low dose of tivantinib may compromise the efficacy of tivantinib for these patients in this meta-analysis. More studies should investigate the efficacy of tivantinib 240 mg for MET-high hepatocellular carcinoma.

Regarding the adverse events in this meta-analysis, tivantinib results in the increase in grade ≥3 neutropenia in MET-high hepatocellular carcinoma but has no obvious in grade ≥3 anemia. Tivantinib at the dose of 240 mg twice daily is not well tolerant for patients, and more methods should be used to control the adverse events. We should consider three shortcomings. Firstly, only three RCTs are involved, and we need more RCTs to confirm these findings. Secondly, there is significant heterogeneity which may result from different durations and doses of tivantinib. Thirdly, the underlying diseases of patients may affect the pooling results.

## 5. Conclusion

Tivantinib may show no obvious improvement in clinical outcomes for MET-high hepatocellular carcinoma.

## Figures and Tables

**Figure 1:** Search and selection of papers.

**Figure 2:** Risk of bias assessment. (a) Authors' judgments about each risk of bias item. (b) Authors' judgments about each risk of bias item presented as percentages.

**Figure 3:** Forest plot for overall survival.

**Figure 4:** Forest plot for progression-free survival.

**Figure 5:** Forest plot for time to progression.

**Figure 6:** Forest plot for grade ≥3 neutropenia.

**Figure 7:** Forest plot for grade ≥3 anemia.

**Table 1:** Baseline data of included studies.

NO Author	Tivantinib group						Control group					
	Number	Age	Female (n)	ECOG status 0/1 (n)	AFP >200 ng/mL	Methods	Number	Age	Female (n)	ECOG status 0/1 (n)	AFP >200 ng/mL	Methods
1 Rimassa 2018 [11]	226	66 (19–87), median (range)	27	141/85	97	Tivantinib 120 mg twice daily	114	65 (26–84)	7	66/48	48	Placebo
2 Kobayashi 2017 [20]	134	—	—	—	—	Tivantinib 120 mg twice daily	61	—	—	—	—	Placebo
3 Santoro 2013 [9]	22	71 (47–83), median (range)	2	16/6	11	Tivantinib 240 mg twice daily	15	69 (46–85)	4	6/9	11	Placebo

## Data Availability

The data sets used and/or analyzed during the present study are available from the corresponding author on reasonable request.

## References

[1] Heimbach J. K., Kulik L. M., Finn R. S. (2018). AASLD guidelines for the treatment of hepatocellular carcinoma. *Hepatology*.

[2] Galle P. R., Forner A., Llovet J. M. (2018). EASL clinical practice guidelines: management of hepatocellular carcinoma. *Journal of Hepatology*.

[3] Bruix J., Reig M., Sherman M. (2016). Evidence-based diagnosis, staging, and treatment of patients with hepatocellular carcinoma. *Gastroenterology*.

[4] Cabibbo G., Enea M., Attanasio M., Bruix J., Craxì A., Cammà C. (2010). A meta‐analysis of survival rates of untreated patients in randomized clinical trials of hepatocellular carcinoma. *Hepatology*.

[5] El-Khoueiry A. B., Sangro B., Yau T. (2017). Nivolumab in patients with advanced hepatocellular carcinoma (CheckMate 040): an open-label, non-comparative, phase 1/2 dose escalation and expansion trial. *Lancet*.

[6] Alves R. C. P., Alves D., Guz B. (2011). Advanced hepatocellular carcinoma. Review of targeted molecular drugs. *Annals of Hepatology*.

[7] Pelosof L., Lemery S., Casak S. (2018). Benefit‐risk summary of regorafenib for the treatment of patients with advanced hepatocellular carcinoma that has progressed on sorafenib. *Oncologist*.

[8] Ueshima K., Nishida N., Kudo M. (2017). Sorafenib-regorafenib sequential therapy in advanced hepatocellular carcinoma: a single-institute experience. *Digestive Diseases*.

[9] Kudo M., Hasegawa K., Chen X.-P. (2016). Regorafenib as second-line systemic therapy may change the treatment strategy and management paradigm for hepatocellular carcinoma. *Liver Cancer*.

[10] Llovet J. M., Ricci S., Mazzaferro V. (2008). Sorafenib in advanced hepatocellular carcinoma. *New England Journal of Medicine*.

[11] Bruix J., Raoul J.-L., Sherman M. (2012). Efficacy and safety of sorafenib in patients with advanced hepatocellular carcinoma: subanalyses of a phase III trial. *Journal of Hepatology*.

[12] Kudo M., Finn R. S., Qin S. (2018). Lenvatinib versus sorafenib in first-line treatment of patients with unresectable hepatocellular carcinoma: a randomised phase 3 non-inferiority trial. *The Lancet*.

[13] Cecchi F., Rabe D. C., Bottaro D. P. (2012). Targeting the HGF/Met signaling pathway in cancer therapy. *Expert Opinion on Therapeutic Targets*.

[14] Gherardi E., Birchmeier W., Birchmeier C., Woude G. V. (2012). Targeting MET in cancer: rationale and progress. *Nature Reviews Cancer*.

[15] Qi X.-S., Guo X.-Z., Han G.-H., Li H.-Y., Chen J. (2015). MET inhibitors for treatment of advanced hepatocellular carcinoma: a review. *World Journal of Gastroenterology*.

[16] Rebouissou S., La Bella T., Rekik S. (2017). Proliferation markers are associated with MET expression in hepatocellular carcinoma and predict tivantinib sensitivity in vitro. *Clinical Cancer Research*.

[17] Munshi N., Jeay S., Li Y. (2010). ARQ 197, a novel and selective inhibitor of the human c-Met receptor tyrosine kinase with antitumor activity. *Molecular Cancer Therapeutics*.

[18] Rimassa L., Abbadessa G., Personeni N. (2016). Tumor and circulating biomarkers in patients with second-line hepatocellular carcinoma from the randomized phase II study with tivantinib. *Oncotarget*.

[19] Matsumoto K., Umitsu M., De Silva D. M., Roy A., Bottaro D. P. (2017). Hepatocyte growth factor/MET in cancer progression and biomarker discovery. *Cancer Science*.

[20] Rimassa L., Assenat E., Peck-Radosavljevic M. (2018). Tivantinib for second-line treatment of MET-high, advanced hepatocellular carcinoma (METIV-HCC): a final analysis of a phase 3, randomised, placebo-controlled study. *The Lancet Oncology*.

[21] Santoro A., Rimassa L., Borbath I. (2013). Tivantinib for second-line treatment of advanced hepatocellular carcinoma: a randomised, placebo-controlled phase 2 study. *The Lancet Oncology*.

[22] Kobayashi S., Ueshima K., Moriguchi M. (2017). JET-HCC: a phase 3 randomized, double-blind, placebo-controlled study of tivantinib as a second-line therapy in patients with c-Met high hepatocellular carcinoma. *Annals of Oncology*.

